# 5G System Overview for Ongoing Smart Applications: Structure, Requirements, and Specifications

**DOI:** 10.1155/2022/2476841

**Published:** 2022-10-11

**Authors:** Hani Attar, Haitham Issa, Jafar Ababneh, Mahdi Abbasi, Ahmed A. A. Solyman, Mohammad Khosravi, Ramy Said Agieb

**Affiliations:** ^1^Departement of Energy Engineering, Zarqa University, Zarqa, Jordan; ^2^Departement of Electrical Engineering, Zarqa University, Zarqa, Jordan; ^3^Abdul Aziz Al Ghurair School of Advanced Computing (ASAC), Luminus Technical University College, Amman, Jordan; ^4^Department of Computer Engineering Engineering Faculty Bu-Ali Sina University, Hamedan, Iran; ^5^Department of Electrical and Electronics Engineering, Faculty of Engineering and Architecture, Nişantaşı University, Istanbul 34398, Turkey; ^6^Department of Computer Engineering, Persian Gulf University, Bushehr, Iran; ^7^Department of Electrical Engineering, Faculty of Engineering, MTI University, Cairo, Egypt

## Abstract

Fifth-generation (5G) cellular networks are state-of-the-art wireless technologies revolutionizing all wireless systems. The fundamental goals of 5G are to increase network capacity, improve data rates, and reduce end-to-end latency. Therefore, 5G can support many devices connected to the Internet and realize the Internet of Things (IoT) vision. Though 5 G provides significant features for mobile wireless networks, some challenges still need to be addressed. Although 5 G offers valuable capabilities for mobile wireless networks, specific issues still need to be resolved. This article thoroughly introduces 5G technology, detailing its needs, infrastructure, features, and difficulties. In addition, it summarizes all the requirements and specifications of the 5G network based on the 3rd Generation Partnership Project (3GPP) Releases 15–17. Finally, this study discusses the key specifications challenges of 5G wireless networks.

## 1. Introduction

The tremendous expansion in mobile connections and innovative applications has raised the demand for new wireless services. This expansion elevates the demands for network technical indicators to be more rigorous. According to Ref. [1], about 20.4 billion Internet of Things (IoT) devices will be connected via machine to machine (M2M) by 2020. According to Ericsson [2], the number of linked devices is predicted to reach 75.4–100 billion by 2025. Meanwhile, according to Huawei, the fifth-generation (5G) subscribers will reach 2.8 billion by 2025 [3].

Furthermore, the emerging 5G technology is the foundation for many future technologies and applications. As a result, the 5G mobile communication system has strengthened at a vital juncture in history to usher in an era of comprehensive information and give a superior user experience. Recently, the industry has been conducting extensive research on crucial 5G technologies, particularly with the emergence of Industry 4.0. As a result, the related inspection, assessment, and verification system must be established and upgraded. With the increasing demand for mobile traffic and the emergence of several technologies that require very high data rates, very low latency, and a broad spectrum, the next generation, 5G, is required to address these issues.

5G technology has eight innovative features such as ultrafast up to 10 Gbps, ultralow latency (1 ms), high capacity (large bandwidth), numerous connected devices, constant availability, and coverage everywhere designed to provide low energy consumption and long battery life [4].

IoT technology is one of the significant drivers of 5G technology. 5G provides innovative infrastructure for the IoT, and IoT use cases that are expected to grow significantly in the future. As a result, the IoT will also make a big difference in communication technology design. While 5 G will bring dramatic changes to cellular systems and the IoT, it faces some significant challenges [5].

The improved massive MIMO technique is another key technology employed in 5G [6]. Employing numerous antennas at the transmitter and/or receive in massive MIMO will considerably improve the wireless system's spectral and energy efficiency [7].

Another approach that allows the antenna to direct radio waves in a particular direction and the receiver is beamforming. Beamforming boosted spectrum efficiency and reduced interference while simultaneously transferring more data from more antennas [8, 9]. Furthermore, recently developed waveforms such as FBMC, UFMC, F-OFDM, and GFDM can overcome pulse shaping, filtering, and precoding issues to reduce the out-of-band (OOB) leakage of OFDM signals [10]. All of these technologies, as well as a few others, are regarded as critical enablers of 5G networks.

However, some issues need to be addressed to implement 5G technology. For example, 5G needs to enable device-to-device communication (D2D) and intelligent vehicle services, provide a reliable network, and ensure privacy and security. While D2D communication improves cellular reuse and interference with femtocells and microcells, and D2D communication can affect system performance because of sharing the same radio resources in the D2D network [11]. In addition, 5G needs to ensure network reliability and availability anytime and anywhere. Security and privacy are two critical challenges that 5G must address. 5G security and privacy challenges increase as the number of users and data exchange increases, increasing the number of threats [12]. In addition, 5G needs to deliver error-free, high-precision data transmission to meet its needs and vision. This is a significant challenge, especially regarding user mobility, which produces a doubly dispersive fading channel that needs complex equalization [13]. All these issues must be addressed efficiently to meet the demand and reach the specific goals of 5G technology.

Several survey papers on 5G technology have been conducted and published in peer-reviewed journals. A comprehensive assessment of the evolution of cellular networks toward 5G networks has been published [14]. The authors emphasized the new architectural paradigm change in radio network layout, air interfaces, smart antennas, cloud, and heterogeneous radio access network design (RAN). They have also detailed the core physical layer technology in detail. Recent research on 5G and IoT has been reviewed in Ref. [15]. They analyzed the new requirements for 5G-enabled IoT. Next, they explained the main methods of 5G IoT and analyzed future IoT issues and trends.

Meanwhile, a study of 5G energy-efficient systems was conducted in Ref. [16]. This paper explored new paradigms, including New Radio (NR), nonorthogonal multiple access (NOMA), machine learning, and cashable networks. Another research study reports energy-efficient scenarios for green communications, such as D2D communications, spectrum sharing, UltraDense networks (UDNs), Massive MIMO, mmWave networks, and IoT [17].

This paper conducts comprehensive research focused on 5G technology. First, the paper outlines 5G networks, including the history of cellular networks, 5G cellular network architectures, 5G service-based architectures, NR 5G technologies, and standalone (SA) and nonstandalone (NSA) modes. Next, this paper will focus on the main requirements and specifications of 5G technology. This includes high data rates, low latency, wide bandwidth, many connected devices, network availability, coverage, low energy consumption, and long life. Finally, 5G specifications challenges such as frequency band completion, large amounts of data, MIMO technology, beamforming, D2D communication, ultralow latency, ultrareliable networks, security, and privacy will be outlined. This paper will help researchers and developers interested in 5G technology understand the challenges of the leading 5G requirements and specifications.

The rest of the paper is structured as follows. Section 2 provides an overview of the 5G system. We reviewed the fundamental requirements of 5G in Section 3, which included the eight 5G enabling critical criteria. Following that, Section 4 outlines the most pressing 5G standard challenges. Finally, Section 5 concludes the paper.

## 2. 5G System Overview

The 5G mobile system is the most recent mobile communication network technology that provides a new way to communicate, including widespread connectivity. Compared to the preceding 1^st^ generation (1G) to the 4th generation (4G), 5G offers much higher performance. Furthermore, 5G should enable a new type of connectivity and applications such as smart vehicles, transport and car communications, and massive video downloads, as media is needed everywhere, a considerable increase in human, IoT interaction, and remote control with haptic feedback, all requires widespread connectivity, as shown in Figure 1.

At the same time, it has been designed to deliver a very low data rate to meet the needs of various applications, such as sensors and IoT applications [18]. In other words, it supports a wide range of applications, from those requiring a low data rate to those requiring a very high data rate with minimal latency. Even though the 5G network initially relied on legacy networks, the 5G cellular architecture is regarded as a heterogeneous network that must comprise macrocells, microcells, picocells, and relays. 5G speed tops out at 10 gigabits per second (Gbps), which is 10 to 100× faster than what you can get with 4G, as shown in Figure 2.

Furthermore, the mobile small cell system is an essential component of the 5G wireless cellular system, which includes both mobile relay and small cell systems.

### 2.1. Architecture of the 5G Cellular Network

It is possible to notice from the existing 5G network that its multiple access methods remain stable, as evidenced by contemporary technologies such as orthogonal frequency-division multiple access (OFDMA), which will most likely be used for the next 50 years [19]. In addition, there is no need to adjust wireless settings from 1G to 4G. However, additional implementation improvements can be made to the base network to meet user criteria [20]. As a result, after the commercial development of 4G is completed, package providers will migrate easily to the 5G network. To address the issues of 5G systems and meet users' needs, developing a 5G wireless cellular architecture requires rapid development. In Ref. [21], most wireless users spent about 80% of their time indoors and 20% outdoors. According to contemporary wireless cellular architecture, an outdoor base station at the cell's center supports outdoor and interior user contact. As a result, the signals would be transferred around the inside walls, allowing interaction between indoor and outdoor users. As a result, significant penetration loss occurs, resulting in a decline in performance due to a fall in spectrum effectiveness and the energy efficacy of wireless communications. To address this challenge, a new design method for building the 5G cellular architecture for various outdoor and indoor scenarios has been developed [22]. Massive MIMO technology [23], which allows for the geographical distribution of tens or hundreds of antenna units, is one of the design strategies that would limit penetration through interior walls. Instead of the conventional MIMO systems that use two or four antennas, massive MIMO systems use big array antenna components that provide significant capacity benefits. For indoor coverage, multiple technologies such as millimeter-wave communication [24], small cells, Wi-Fi, ultrawideband [25], and visible light communication [26] are suitable for short-range, high data rate responses. However, visible light and millimeter-wave responses require the utilization of higher frequencies, which are not typically used in cellular responses. Notably, long-distance and external deployment of these high-frequency waves is not advised because the waves would not successfully penetrate dense materials.

On the other hand, these waves might be efficiently disseminated by flora, gases, and raindrops. Millimeter-wave and visible light responses have a wide bandwidth and can increase the data transmission rate of indoor setups [27]. In addition to the emergence of new spectra that are generally not used for radio interactions, another approach to solving the problem of spectrum shortages is to use cognitive radio (CR) networks to improve the spectral utilization of new radio spectra [28]. The heterogeneity of 5G cellular architectures requires the integration of relays, small cells, microcells, and macrocells.

In particular, the mobile small cell idea is a crucial component of the 5G wireless cellular network, which comprises small cell concepts and mobile relays [29]. This concept was developed to preserve users' connectivity with significant mobility in high-speed trains and vehicles. Furthermore, mobile small cells are installed inside moving vehicles to connect with users, while the massive MIMO unit is installed on the vehicle's exterior to communicate with the outdoor base station. From the user's point of view, the mobile small cell is identified as a regular base station, and the associated user is identified as a single entity with a base station, indicating the separation of indoor and outdoor construction. Furthermore, small mobile cell users employ high data rates for bandwidth-intensive services while reducing signaling overhead. The 5 G wireless cellular network design has two logical layers: network cloud and radio network [30].

Different elements with different functions make up a wireless network. The network functions virtualization (NFV) cloud comprises a control plane entity (CPE) and a user plane entity (UPE), with the more critical utility of the planes associated with the control plane and user plane, respectively.

Notably, the 5G cellular network architecture is critical in both the backhaul and front-end networks.  Figure 3 shows a multilayer network with macrocells covered by D2D links, femtocells, picocells, and relays. Implementing multiple layers in a cellular network architecture results in the excellent management of interlayer and intralayer interference, resulting in improved overall power consumption, spectral efficiency, coverage, and capacity.

### 2.2. New Radio 5G Technology

The 3GPP is in the process of defining a new 5G radio interface known as NR [31]. Enhanced Mobile Broadband (eMBB) will remain substantial, driving demand for increased system capacity, enhanced coverage, and faster data rates. Nonetheless, the ambitions of 5G transcend beyond eMBB. For example, MMTC, often known as IoT, is concerned with enabling meager device cost and energy consumption, offering extreme coverage, and handling a massive number of devices.

Another 5G goal is Ultra-Reliable Low-Latency Communication (URLLC), which provides data delivery with very low latency, for example, addressing critical industry applications. Furthermore, it is feasible that new and unexpected use cases will emerge during the life of NR. As a result, forward compatibility, which allows for the easy implementation of future optimizations, is a critical design requirement. Furthermore, improved network energy performance than the current systems is a key principle.  Figure 4 depicts the several critical technologies that NR will support in 5G [32].

### 2.3. Standalone and Nonstandalone Mode

To improve 5G end-to-end performance, multiconnectivity is the optimal solution that combines long-term evolution (LTE) with reliable sub-6 GHz connections, such as simultaneous millimeter-wave connections. It can be used in the NSA mode with 5G NR [33]. This means that the 5G NR NSA mode means that the 4G network is used to connect to the control plane, and the 5G NR network is dedicated to the user plane. In contrast, in the standalone (SA) mode, both the control plane and the user plane use only the 5G NR leading network.  Figure 5 shows both standalone and nonstandalone 5G NR systems. Technical work on NR began in the spring of 2016. The first release was part of Release 15 of 3GPP, and the NR specification was completed in late 2017. This initial release is limited to nonstandalone NR operations. NR devices rely on LTE for the initial access and mobility [34]. In addition, standalone NR operations are supported in the final release of 15 specifications available after June 2018 [35]. The difference between standalone and nonstandalone operations is primarily related to interface issues to the upper layers and core networks. The basic wireless technology is the same in both cases.

## 3. 5G Requirements

5G technology is driven by eight specification requirements, as shown in Figure 6:

- 100% coverage
- Up to 10 Gbps data rate—>10 to 100x speed improvement over 4G and 4.5 G networks
- one-millisecond latency
- 1000 × bandwidth per unit area
- Up to 100x number of connected devices per unit area (compared with 4G LTE)
- 99.999% availability
- 90% reduction in network energy usage
- Up to 10-year battery life for the low-power IoT device

### 3.1. High Coverage

Another issue for which 5G is looking for answers is coverage. 5G necessitates the perception of complete coverage [36]. By providing adequate coverage, technologies like IoT, D2D, and V2V can connect with the network from any location. Furthermore, because 5G enables network availability of up to 99.999 percent and coverage of nearly 100 percent, various services, including the technologies mentioned above, will be able to access the network at all times and from any location.

### 3.2. High Data Rate

The massive expansion in mobile connections over the last few years has increased the demand for large data volumes. This is the primary driving force behind the need for a high data rate in 5G technology. The 5 G technology will support many services and applications that require high data rates. This system is designed to boost data rates up to 10 Gbps, a 10-fold improvement over the 4G network. Several advanced technical solutions, such as mmWave, massive MIMO, and various modulation and coding methods, enable 5G technology to achieve this goal [37].

### 3.3. Substantially Low Latency

One of the most significant needs that 5G focuses on is providing very low latency, where latency is the amount of time it takes for a request to complete an end-to-end round trip or the time it takes for the network to respond [38]. 5G latency will be significantly reduced to 1 ms end-to-end round trip. The end-to-end round trip delay latency of a 5G network is ten times lower than that of a 4G network [39]. The low latency of 5G will enable various applications, such as AR, VR, self-driving cars, and remote surgery. [40].

### 3.4. Wider Bandwidth

Increasing capacity causes an increase in bandwidth. The traditional LTE network operates on a frequency band of 3 GHz. This property restricts 5 Gbps implementations and complicates the design difficulty [41]. A high bandwidth per unit space enables a large number of linked devices in a small area. This is possible using mmWave technology [42]. 5G technology will give 1000 times the bandwidth per unit area while increasing capacity by up to 10 Gbps [43].

### 3.5. Massive Number of Connected Devices

Another significant aim of the 5G system is dramatically expanding capacity and enabling a massive number of concurrently connected devices. Compared to legacy systems, 5G will support up to 10–100 times the number of concurrently connected devices [44]. Massive IoT devices and sensors will be connected to the 5G network because it is a crucial infrastructure network for IoT. However, the communication channels must also ensure a very high data throughput and minimal latency. Although connecting billions of devices and sensors to the network simultaneously is difficult, this goal can be realized by utilizing solutions like massive MIMO, D2D technology, and cloud RAN [45].

### 3.6. High Availability

Many of the services and applications enabled by the 5G network necessitate constant network connectivity. As a result, 5G promises to deliver a perception of 99.999 percent availability, implying that the network will always be operational. This functionality would enable users and devices to connect to and access the network at any time [46].

### 3.7. Enhanced Battery Life

The battery life in 5G is expected to be 10 years. This goal is attainable with the advancement of battery technology and power-consuming electronics. Increasing battery life is critical for devices with limited battery capacities, such as laptops, cellphones, and tablets [47].

### 3.8. Low Energy Usage

5G will lower network energy consumption by up to 90%. This reduction in energy consumption by 5G must occur as it provides extraordinarily high speed [31, 48]. Even though 5G provides fast data rates, low latency and coverage, and 99.999 percent availability, it will increase energy consumption by allowing rapid switching between sleep and active modes.

## 4. 5G Specifications Challenges

Because of the high demand and complex features of 5G networks, various technological challenges must be addressed.

### 4.1. Wide Frequency Bands

Network traffic and required data rates will increase in the future. These developments require a higher frequency band than that used in LTE systems. Therefore, the current frequency band with a range below 4 GHz cannot support 5G requirements. Therefore, we need new technologies that can support high traffic and data rates anywhere, under any conditions. Millimeter-wave technology is the best way to meet such needs at the same time. This is because mmWave provides wider frequency bands supporting 5G network traffic data.

Moreover, using the mmWave with massive MIMO and beamforming techniques presents suitable 5G network implementation options. However, supporting high traffic and additional frequency bands increase system complexity and thus make the 5G network application challenging. More issues of wide frequency bands are coverage limitation and higher attenuation compared to the low-frequency bands [49].

### 4.2. Huge Data Volume

Each year, the number of devices linked to the Internet grows considerably, as does the volume of data. The major challenge with 5G is the billions of gadgets and sensors connected to the Internet. According to Huawei and Information Handling Services (IHS) forecasts [50], the number of linked devices will reach 75–100 billion by 2025. As a result, 5G must be capable of handling vast amounts of data from an enormous number of connected devices and sensors and processing it concisely [51]. As data volume grows, it causes difficulty and complexity in securing, processing, regulating, and analyzing massive amounts of data [52].

### 4.3. Ultralow Latency

Providing an ultralow latency carrier is a severe situation confronted via way of means of 5G systems. Many crucial packages, including self-using and healthcare enterprise uses, require latencies of 1 ms. To offer an extensively low latency under 1 ms with huge statistics is a complicated challenge that 5G has to achieve. Besides that, machine-type communications (MTC) is a utility that 5G networks in all likelihood want to aid wherein the gadgets mechanically speak with every other possibility [53, 54]. For applications such as V2V communication, this type of communication requires very low latency. The METIS and METIS-II projects, which are European projects for traffic safety, and the “connected cars” use case addresses information exchange among vehicles and with the infrastructure to enable those as follows:

- A safer and more efficient transportation
- Real-time remote computing for mobile terminals.

On the other hand, it has been proposed that traffic efficiency and safety be a typical application test case, with latency being critical in system evaluation. Intelligent traffic systems are a common scenario shown in METIS and METIS-II, in which cars require fast data sharing to avoid accidents. Low latency will also improve user experience in applications such as multiuser gaming. This reduction in latency necessitates technological innovation in waveform design and flexible architecture in the network's higher layers, both of which can be met by wireless software-defined networking. [55, 56].

### 4.4. Ultrareliable Network

The accuracy of data transmission without errors is known as reliability. Several future applications and services will want highly dependable networks that will not tolerate failures. Operating at high frequencies using mmWave, 5G will make wireless technologies more vulnerable. As a result, 5G must address this difficulty by utilizing technologies such as beamforming, MIMO, and software-defined networking (SDN) [57].

### 4.5. Security and Privacy

In wireless communication systems, security and privacy are two of the most critical considerations. They are also the two most significant problems for the 5G system. 5G will accommodate many connected devices with fast data rates and massive capacity, raising security and privacy concerns. As a result, 5G must provide and guarantee end-to-end privacy and security for users. The vast number of connected devices to the 5G network with massive amounts of data and security and privacy concerns were two of the critical issues that 5G faced. To protect data and users' privacy, security and privacy must be considered [58, 59].

### 4.6. Smart Automobiles

Once 5G is built, self-driving automobiles and smart automobile technologies will be available. Smart cities are also projected to be launched to support this application. 5G will enable smart vehicles to connect and serve as a data transfer hub for communication with roadside infrastructure and other services [60]. Because of safety-critical use cases and rapidly changing vehicular network architecture, enabling smart automotive technologies necessitates networks with significantly reduced latency and exceptionally high dependability [13]. As a result, the 5G network must be designed to meet the rigorous QoS requirements of smart vehicle systems [54].

### 4.7. Spectrum Availability

The frequency spectrum is rare and is currently a supersaturated product. Therefore, it is important to evaluate the availability of the spectrum. Existing mobile technologies use frequencies ranging from 300 MHz to 3 GHz [61]. Regardless of this, new 5G frequency bands are being investigated. 5G uses low and high frequencies, as well as very high frequencies. Low frequencies (<1 GHz) and high frequencies (1–6 GHz) are commonly used for mobile communications. On the other hand, very high frequencies (30–300 GHz) represent a new spectral option for 5G. In Europe, Japan, South Korea, and the United States, intervals between 3.5 and 4.5, and also 28 GHz include targeted or allocated licensed and unlicensed bands. In addition, the 39 GHz band is typically used for 5G in the United States and Canada. The 39 GHz band can be helpful as this bandwidth is unsaturated and therefore is available for mobile communications.  Figure 7 shows 5G radio frequency spectrum [62].

### 4.8. Air Interface

Due to the exacting requirements of 5G, a new air interface must be developed. Thus, new air interfaces, known as NR, are being created according to modulation schemes, which are being developed based on the scope of future mobile communication systems [63] since 5G using mmWaves technology, having small wavelengths, will require small antenna sizes. In other words, 5G uses a massive of small antennas. Exploiting beamforming technology directs the antenna's signals into a specific and desired direction, enhances the data rate, and increases the signal strengths with low interference [64]. However, 5G must overcome hardware design challenges, power consumption, directional accuracy, and analog-digital and digital-analog processes [65].

### 4.9. Special Protocols Adapt with 5G

Recent research is directed to apply particular protocols to improve the 5G wireless network specifications, such as the data rate, network congestion, and security. Applying network coding, co-operation networks, hybrid networks, etc. is an important technique to achieve the desired improvement.

Accordingly, applying network coding and co-operation networks resulted in what is called co-operation network coding (CoNC), which resulted in improving the data rate, network congestion, security, transmission packet error rate (PER), and bit error rate (BER) [66–69], where [51] the hybrid network was applied to improve the transmission range and to improve the PER. Moreover, improving the application over the physical layer was widely proposed [70–72], and 5G applications more and more cover medical fields.

Future work is planned so as to focus on viewing an inclusive article that accumulates information for the medical applications that are suggested for 5G and B5G based on our published work in [73–77].

## 5. Conclusion

A complete survey of 5G technologies requirements and specifications challenges has been undertaken in this study. The survey describes the overall network architecture and essential requirements for the 5G network. Meanwhile, the paper introduced technologies that would make 5G a reality, including mmWave, massive MIMO, beamforming techniques, and other advanced technologies. Finally, the study outlined several essential difficulties that must be effectively solved before 5G technology can be globalized. This survey paper provides readers with a concise and in-depth review of 5G wireless networks.

## Figures and Tables

**Figure 1:** 5G use cases.

**Figure 2:** Comparison between 3G, 4G, and 5G data rates.

**Figure 3:** 5G cellular network architecture.

**Figure 4:** Technologies supported by 5G NR.

**Figure 5:** Nonstandalone 5G NR and standalone 5G NR.

**Figure 6:** Specification requirements for 5G technology.

**Figure 7:** 5G radio frequency spectrum.

## Data Availability

The experimental data used to support the findings of this study are available from the corresponding author upon request.
